This article has been retracted.

# Phase 2 Assessment of a New Functional Pain Scale by Comparing It to Traditional Pain Scales

**DOI:** 10.7759/cureus.24522

**Published:** 2022-04-27

**Authors:** Harris W Thomas, Adeolu A Adeboye, Rachel Hart, Harshavardhan Senapathi, Michael Hsu, Sneha Singh, Tejaswini Maganti, Victor Kolade, Abistanand Ankam, Amlish Gondal

**Affiliations:** 1 Pain Management, Guthrie Robert Packer Hospital, Sayre, USA; 2 General Surgery, Guthrie Robert Packer Hospital, Sayre, USA; 3 Trauma and Acute Care Surgery, Guthrie Robert Packer Hospital, Sayre, USA; 4 Anesthesia, Guthrie Robert Packer Hospital, Sayre, USA; 5 Internal Medicine, Guthrie Robert Packer Hospital, Sayre, USA

**Keywords:** patient safety, objective pain assessment, patient reported experience, functional pain scale, pain rating

## Abstract

Background

Assessment of pain has always been subjective and is commonly assessed using a numeric pain scale (NPS) or Wong-Baker faces scale. The pain intensity score is not standardized and relies on individuals’ past experiences. The disadvantage of using such pain assessment scales and treating the numbers can lead to overdosing on analgesics leading to unwanted side effects. The Robert Packer Hospital/Functional Pain Scale (RPH/FPS) was developed as a tool for the objective assessment of pain and its impact on a patient’s function.

Aim

The study aimed to validate the RPH/FPS scale against NPS and Wong-Baker faces scale in medical, surgical, and trauma patients. The patients’ were also asked to rank the scales as one (1) being the most preferred to three (3) being the least preferred.

Design

This prospective, observational cohort study compares the two most common pain scales, the NPS and the Wong-Baker Faces, to the RPH/FPS.

Methods

Spearman correlation was used to test for correlation between the three scales, and Wilcoxon rank-sum test was used to compare means between the RPH/FPS and NPS. The study participants were also asked to rate their preferences for the scales by rating the most preferred of the three scales as one (1) and the least preferred number three (3).

Results

The RPH/FPS had a strong correlation with both the NPS and Wong-Baker Faces scales (RPH/FPS vs. NPS R=0.69, p<0.001: RPH-FPS vs. Wong-Baker Faces R=0.69, P<0.001). As for preferences, the RPH/FPS was ranked first on 36.9% of the surveys followed by NPS on 35.9%, and the Wong-Baker Faces on 22.3%. There were 4.9% of the surveys missing the preference rankings.

Conclusion

The results validate the RPH/FPS scale against the NPS and Wong-Baker Faces scales. This gives the clinicians a tool for objective assessment of pain and its effect on the recovery process, thereby minimizing the observed disconnect that sometimes happens between the reported pain intensity* *level and the providers' observation of the patient.

## Introduction

Pain is defined according to the International Association for the Study of Pain (IASP) as "an unpleasant sensory and emotional experience associated with actual or potential tissue damage or described in terms of such damage" [1].

Pain is a subjective assessment determined primarily by a patient's self-report [2]. Two of the most common pain assessment tools used are the numeric pain scale (NPS), and the Wong-Baker Faces pain scale. The difficulty with monitoring and medicating according to pain intensity is that it has a direct correlation with experiences. A person who has had more painful experiences, either chronic or acute pain, may report their pain intensity level lower than a person with fewer pain experiences. There are additional factors that may contribute to the difficulty in recording pain, including gender and culture. The patient self-report may also have a provider and patient disconnect, where the provider observes behaviors that would normally be considered comfortable by a patient. 

The NPS and Wong-Baker Faces scales have been used for many years and validated many times [3]. However, the need for a new type of pain scale has been recognized, and several have been developed in the recent past [4-6]. The hope is that the RPH/FPS [7] will replace the NPS and Wong-Baker Faces scales. The RPH/FPS was designed to clarify the effect of pain on three areas of recovery; sleep, ability to complete activities of daily living (ADLs), and concentration. The RPH/FPS still has a numeric component but also uses descriptive words to describe the patient's pain effect. This new scale helps bridge the gap that the pain intensity scales can open and define how both patient and provider interpret pain.

The aim of the phase 2 study was to validate this scale for general surgery, trauma, and internal medicine patients that have not seen the RPH/FPS scale prior to this admission. Our study shows a comparative data analysis of the RPH/FPS to NPS and Wong-Baker Faces scales. Implementing the RPH/FPS into the electronic medical records (EMR) should aid the providers in having a complete assessment of the patient and improve the patient experience.

## Materials and methods

Patient population

In accordance with institutional guidelines, Institutional Review Board approval (IRB#2007-51) was obtained prior to initiating the current study. All patients were prospectively enrolled in the observational cohort study after obtaining verbal informed consent. Inclusion criteria were set as adult patients with inpatient admittance. Exclusion criteria were set as <18 years of age, a prior diagnosis of cognitive impairment, a history of opioid abuse, and non-English speakers. All patients were identified through a daily admission report prospectively enrolled for this study without any changes to their quality of care if they refused to participate.

Data collection

For the purposes of the study, patient demographics and characteristics of hospitalization were collected, including age, gender, education, admitting service, and diagnosis. Patients were also asked to complete three separate health questionnaires that evaluated their pain. These questionnaires included the NPS, Wong-Baker Faces pain scale [8], and the RPH/FPS.

The NPS evaluates a patient's subjective pain level based on a scale of 0-10, with 10 being the worst pain and 0 being no pain at all. The Wong-Baker Faces scale was originally developed for the evaluation of pediatric patient scales but has since been used internationally for patients >3 years of age to evaluate their pain. The scale asks patients to evaluate their pain level based on a set of different faces associated with an objective number 0-10 (Figure 1). The RPH/FPS is a recently developed functional pain score that aims to evaluate pain on a more objective scale by prompting how pain affects a patient's daily activities (Table 1). The scale is used by asking four questions to the patient. The first question is "Are you having pain right now?" The second is asking how pain affects the patient's sleep, i.e., "are you able to sleep, is it slightly affected, or are you unable to sleep because of pain?" The third question then moves to the patient's ability to complete activities of daily living, i.e., are they able to get out of bed by themselves, do they need assistance, or are they able to participate in physical therapy (PT) and occupational therapy (OT)? Finally, the last question is how is pain affecting their concentration? Are they able to use distractions like watching TV, listening to music, or carrying on a conversation with a visitor? These are examples of passive distractions. Active distractions might be considered doing a puzzle, playing a game on their phone, coloring, and doing crafts. The healthcare team member can then take the answers and determine the appropriate pain number and the determined medication and dose by the pain scale. To further assess the validity of the RPH/FPS against the NPS and Wong-Baker Faces, both patients and administrators of surveys completed a prompt asking their preference on the pain scale.

**Figure 1:** Wong-Baker Faces pain scale.

**Table 1:** Robert Packer Hospital/Functional Pain Scale.

Descriptor	Definition
No Pain (0)	No pain
Minimal (1)	Hardly noticeable/No impact on ADLs/Sleep not affected and able to use passive distraction for comfort. Mild range order.
Mild (2)	Noticeable when not distracted/No impact on ADLs/Sleep only slightly affected and able to use both passive and active distraction for comfort. Mild range order.
Uncomfortable (3)	Pain is present but can complete all ADLs/ Sleep is slightly affected and passive distraction only gives marginal relief. Mild range order.
Moderate (4)	Constantly aware of pain but can complete ADLs with modification/ Sleep marginally affected at times/Passive distraction is of no use, but active distraction gives some relief. Moderate range order.
Distracting (5)	Aware of pain/ Able to complete some ADLs but limited by pain/ Sleep is affected and active distractions are only slightly useful. Moderate range order.
Distressing (6)	Pain is present/ Unable to complete most ADLs limited by pain/Sleep is difficult and active distraction is only marginal. Moderate range order.
Unmanageable (7)	Pain interferes with normal ADL/ Nothing seems to help/Sleep is very difficult/ Active distractions are very difficult to concentrate on. Severe range order.
Intense (8)	Cannot complete any ADLs without much assistance/ Can’t concentrate/Conversation is difficult/Unable to sleep and unable to use a distraction. Severe range order.
Severe (9)	Cannot do any ADLs even with assistance, can barely talk/unable to sleep, and unable to use a distraction. Severe range order.
Immobilizing (10)	Unable to move or talk due to intensity of pain/ Unable to sleep and unable to use a distraction. Severe range order.

Statistical analysis

A power analysis using the two means equations in the Power and Sample Size Calculation program [9] was performed to determine the appropriate sample size with the assumption of a standardized response mean of 0.29 for the RPH/FPS, a power of 0.80, error rate of 0.05, and estimated loss to follow-up rate of 0.10. Summary statistics were performed for the demographics and hospitalization characteristics of the study cohort. Additionally, summary statistics were performed to determine the preference of the pain scale of the study cohort. Any differences in scores between types of pain questionnaires were evaluated using a Wilcoxon rank-sum test. Convergent validity (Table 2) of the RPH/FPS was evaluated using Spearman's correlation analysis, and the strength of correlation was categorized using the following cutoffs: weak (|r| < 0.3). All statistical tests were performed using RStudio (RStudio, PBC, Boston, MA) using an alpha value of 0.05.

**Table 2:** Phase 2 convergent validity on three pain scales. RPH/FPS: Robert Packer Hospital/Functional Pain Scale; NPS: Numerical pain scale.

Pain scale	r	p-value
RPH/FPS vs. NPS	r=0.68	p<0.001
RPH/FPS vs. Wong-Baker Faces	r=0.69	p<0.001
Wong-Baker Faces vs. NPS	r=0.82	p<0.001

## Results

Study cohort

Based on the N from the pilot study, it was calculated that 103 patients were eligible for this study. After inclusion and exclusion criteria were applied, the final study cohort consisted of 101 patients. The mean age was 64.4 years, with 59.4% being male. Patients were admitted under the primary services of trauma, surgery, and internal medicine. There were eight trauma patients (7.9%), 13 surgical patients (12.8%), and 80 internal medicine patients (79.2%).

Convergent validity

Patients reported a mean NPS score of 7.75 ± 2.03, a mean Wong-Baker Faces score of 7.77 ± 2.01, and a mean RPH/FPS score of 6.08 ± 2.37 (Table 3). Although it appears that the RPH/FPS is showing a lower score than the self-report, the score was deemed to be statistically insignificant. Spearman's correlation analysis demonstrated a strong correlation between the RPH/FPS and NPS scale (r=0.69; p<0.001). A similar result was observed when comparing the RPH/FPS and Wong-Baker Faces score (r=0.69; p<0.001) as well as the Wong-Baker Faces and NPS scale (r=0.82; p<0.001).

**Table 3:** Phase 2 patient characteristics. Faces: Wong-Baker Faces Pain Scale; NPS: Numerical pain scale; RPH/FPS: Robert Packer Hospital/Functional Pain Scale.

Patient characteristics	N (%)	Mean (SD)	Median (Range)
Age	101 (99%)	64.4 (14.6)	65.5 (21-88)
Faces score	101 (100%)	7.77 (2.01)	8 (2-10)
NPS score	101 (99%)	7.75 (2.03)	8 (1-10)
RPH/FPS score	101 (99%)	6.08 (2.37)	6 (1-10)

The RPH/FPS scale was ranked the highest in terms of preference by 36.9% of the study cohort. Comparatively, NPS was ranked the highest in preference by 35.9% of the cohort, and FACES was ranked the highest by only 22.3% of patients. A total of five individuals (4.8%) did not complete the preference survey (Table 4). Further analysis demonstrated that 23.1% of patients had a preference of RPH/FPS > NPS > FACES whereas 13.5% of patients preferred RPH/FPS > FACES > NPS. When NPS was rated highest, 21.2% of patients preferred the order of NPS > RPH/FPS > FACES and 15.4% preferred NPS > FACES > RPH/FPS. Lastly, when FACES was preferred, 12.5% ranked their preference as FACES > RPH/FPS > NPS, and 9.6% of the study cohort ranked their preference as FACES > NPS > RPH/FPS (Table 5).

**Table 4:** Phase 2 patient preferences. RPH/FPS: Robert Packer Hospital/Functional Pain Scale; NPS: Numerical pain scale; Faces: Wong-Baker Faces Pain Scale

Variable	N = 103
Age	
Mean (SD)	64.4 (14.6)
Median	65.2 [21.0, 88.0]
Missing	1 (1.0%)
RPH/FPS	
Mean (SD)	6.08 (2.37)
Median [Min, Max]	6.00 [ 1.0, 10.0]
Missing	1 (1.0%)
NPS	
Mean (SD)	7.75 (2.03)
Median [Min, Max]	8.0 [1.0, 10.0]
Missing	1 (1.0%)
Faces	
Mean (SD)	7.77 (2.01)
Median [Min, Max]	8.0 [2.0, 10.0]
Missing	0 (0%)
Patient preference	
RPH/FPS	38 (36.9%)
NPS	37 (35.9%)
Faces	23 (22.3%)
Missing	5 (4.9%)

**Table 5:** Order of patient preferences. RPH/FPS: Robert Packer Hospital/Functional Pain Scale, NPS: Numerical pain scale, Faces: Wong-Baker Faces Pain Scale.

Order of preferences 1-3	Patient choice of order	% of top preference
RPH/FPS; NPS; Faces	24	23.30%
RPH/FPS; Faces; NPS	14	13.60%
NPS; RPH/FPS; Faces	22	21.40%
NPS; Faces; RPH/FPS	15	14.60%
Faces; RPH/FPS; NPS	13	12.60%
Faces; NPS; RPH/FPS	10	9.70%
Missing preference	5	4.90%

## Discussion

The practice of dosing to a unidimensional pain intensity number such as the NPS was once the most accepted. The main problem with this practice is that there has been no research completed to determine a perfect dosage for each range of pain scores, i.e., 1-3 out of 10 considered mild, 4-6 out of 10 moderate, and 7-10 out of 10 being severe [10]. Also, it is not always appropriate to dose according to those numbers without knowing the person's opioid tolerance or history of pain and medications. Pain is a subjective experience; pain intensity is determined by the person experiencing the pain and is often obtained through the use of a pain intensity scale. The task of assessing pain is difficult; there is no objective data such as vital signs to determine pain intensity [11]. Therefore, monitoring how pain affects the patient's response to pain by observing sleep, ability to function, and concentration levels are appropriate measures to manage the pain.

Using the RPH-FPS would be safer for the patient experiencing pain as well. By using this scale versus the NPS or Wong-Baker FACES scales, there should be less chance of an adverse event. The first premise in all areas of healthcare is "Do no harm" [12]. Dosing to a number can put the patient at risk of respiratory depression if they say their pain intensity level is higher than what the RPH-FPS scale observed. It has also been reported that The Joint Commission (TJC) and the Centers for Medicaid and Medicare Services (CMS) are critical of the practice of dosing to a number or range orders. The belief is that this practice does not individualize medications for a specific patient [13]. The American Society for Pain Management Nursing (ASPMN) position statement is very clear on the TJC focus of their pain standards. The statement reads, "Since the release of TJC pain standards, pain experts and others have questioned the safety and efficacy of focusing on pain intensity as the primary, and sometimes only, element of pain assessment [11,14-20]. Most of the concerns focused on an observed increase in opioid-related adverse events, many of which involved the administration of opioid doses based solely on pain intensity. In 2016 The American Pain Society published a set of guidelines on postoperative pain management [5]. This was a collaborative paper with several organizations meeting and making the recommendations. The guidelines have several recommendations involving education, individualized treatment plans, assessment for adverse events, and assessment tools. The guidelines recommendation regarding assessment was listed as a strong recommendation, but low-quality evidence. The guidelines emphasize self-report, but they also insist that a validated pain scale be used.

The purpose of the study was to validate a new functional pain scale that might give the healthcare team an objective tool to manage pain [21]. The results show that the RPH-FPS is a validated scale compared to the NPS and the Wong-Baker FACES scales. The patient preference was also shown to favor the new scale. This scale improves communication between the healthcare team and the patient.

There are a few functional pain scales being used today [13], but the nurse or physician has to document using the pain intensity score. None of the scales are based on a 1-10 pain score. The Clinically Aligned Pain Assessment (CAPA) asks questions about comfort, change in pain, pain control, functioning, and sleep but ultimately depends on a score based on the NPS [21]. The scale that was introduced by the Salem Healthcare in Salem, Oregon, uses an analog scale and looks like a thermometer with descriptive words where the numbers would be. One of the first functional pain scales uses a combination of Wong-Baker FACES, NPS, descriptive words, and reporting pain at rest and with activity [10]. The RPH/FPS is meant to replace the 0-10 scale by defining what those numbers mean as they relate to how pain is affecting sleep, activities, and concentration.

Although the RPH/FPS appears to be a tool that the healthcare team can use to objectively assess and communicate with the patient, there may be shortcomings to the scale. First, the scale was supposed to be at a fourth-grade reading level; however, it may take additional discussion between the physician or nurse doing the assessment and the patient due to not knowing the patient's cognitive ability. The descriptive words and definitions of each might seem too complex for some patients. Finally, the RPH/FPS scale may not be the most beneficial in some clinic offices, EDs, or recovery units after a procedure or surgery.

In spite of these few examples of where it would not work or be beneficial, the RPH/FPS is an overall good, validated scale. It will encourage more conversation between the healthcare team and the patient regarding pain and opportunities to explore non-pharmacologic means of pain control. It will also create more chances for healthcare providers to discuss medications, what to avoid, and what is safe for the patient. Finally, this scale gives the healthcare provider a tool that eliminates the possible disconnects between what they observe and the pain intensity score that the patient might report.

This was a randomized trial, and it is acknowledged that the demographics are heavily skewed towards internal medicine patients. With this in mind, additional studies may have to be completed to validate this scale in trauma and general surgery areas. Additionally, additional studies may be completed in specialty clinic settings to see the effectiveness of this type of assessment.

## Conclusions

The RPH/FPS allows hospital-based clinicians to expand past numerical scores and facial expressions to assess the level of disruption that pain imposes on patients. The RPH/FPS can be used by auxiliary services such as physical therapy and occupational therapy (PT/OT) to glean information about how pain affects function. The care coordinator will also be able to find helpful information regarding the patient's ability to concentrate due to pain, i.e., "Is now a good time to discuss POC, or is the patient unable to concentrate due to pain." Auxiliary services are unable to find any of this information using the NPS or any other unidimensional pain scale. Further studies should expand the population in which the RPH/FPS is tested and compared to existing pain scales.
